# The suppressing role of miR-622 in renal cell carcinoma progression by down-regulation of CCL18/MAPK signal pathway

This article has been retracted.

**DOI:** 10.1186/s13578-018-0212-8

**Published:** 2018-03-02

**Authors:** Tian Li, Xiangzhou Sun, Kewei Xu

**Affiliations:** 1 Department of Urology, The Fifth Affiliated Hospital of Guangzhou Medical University, 621 Gangwan RD, Huangpu District, Guangzhou, 510700 Guangdong China; 2 Minimally Invasive Technique and Product Translational Center, Guangzhou Medical University, Guangzhou, Guangdong China; 3 Department of Urology, The First Affiliated Hospital of Sun Yat-Sen University, Guangzhou, Guangdong China; 4 Department of Urology, The Second Affiliated Hospital of Sun Yat-Sen University, Guangzhou, Guangdong China

**Keywords:** miR-622, Kidney cancer, CCL18, MAPK

## Abstract

**Background:**

MicroRNAs have emerged as critical modulators of carcinogenesis and tumor progression including renal cell carcinoma (RCC). MiR-622 plays as a tumor inhibitor in some types of cancer, however, its role in kidney cancer is unknown. The purpose of the present work is to investigate the functional behaviors and regulatory mechanism of miR-622 in RCC.

**Results:**

We examined the expression of miR-622 in RCC and adjacent normal tissues and then explored the roles of miR-622. The results of this analysis indicated that miR-622 activity was significantly downregulated in RCC tissues compared with the corresponding normal tissues, so did in RCC cell lines. MiR-622 was associated with RCC aggressiveness. MiR-622 in RCC cells decreased CCL18 expression and suppressed CCL18 activated MAPK signal pathway. Using Western blot and luciferase reporter assays, it was verified that CCL18 was a direct target of miR-622. A specific and inverse correlation between miR-622 and CCL18 expression was found in human RCC samples.

**Conclusions:**

The results demonstrated that miR-622 acted as a tumor-promoting miRNA by targeting CCL18 in RCC.

## Background

Renal cell carcinoma (RCC) is the most common type of human kidney cancer, and clear cell RCC (ccRCC) is one of major histologic subtype. There is a rapid rise in the incidence of (RCC) [1, 2]. When RCC patients are diagnosed, about 1/3 of RCC patients have metastasis [2]. Therefore, it is very important to find new molecular biomarkers in early stage of RCC patients or new targets to guide RCC diagnosis or therapy. Genetic biomarkers for RCC have been widely investigated including microRNAs (miRNAs).

MiRNAs are a class of noncoding RNAs with about 22 nucleotides in length. MiRNAs have been recognized as key regulators of gene expression at the post-transcriptional levels by their direct interaction with the 3′-UTR of complementary mRNA target transcripts, which facilitates their degradation or inhibits their translation [3–5]. They are broadly involved in a variety of biological functions of RCC development and progression including cell proliferation, metastasis, angiogenesis, drug resistance, metabolism and others [4–6]. MiR-622 plays an inhibiting role in various cancer like glioma [7], colorectal cancer [8–10], hepatocellular carcinoma [11, 12], lung cancer [13], esophageal squamous cell carcinoma [14] and gastric cancer [15]. The biological functions of miR-622 in the reported cancers include cell proliferation and metastasis [7–15]. But, the regulatory mechanism of miR-622 in RCC is still unknown.

In this study, we attempted to characterize the molecular mechanisms of miR-622 in RCC in order to explore new potential therapeutic method. We performed a series of tests and found consistently lower expression levels of miR-622 in kidney cancer cells. MiR-622 could lead to the suppression of cell proliferation and metastasis of kidney cancer. It was verified that CCL18 was a target gene of miR-622 in kidney cancer cells, which was from the prediction result. The clinical results demonstrated that miR-622 was negatively associated with CCL18 in the samples of RCC patients. The further investigation indicated that miR-622 suppressed CCL18 activated MAPK signal pathway in RCC cells.

## Methods

### Samples

Kidney cancer samples and their matched normal adjacent tissues were gained from patients. The diagnosis was based on the pathological evidence. The samples were collected and stored at − 80 °C. All samples were collected after the patients provided the written informed consents from the Ethics Board of the Fifth Affiliated Hospital of Guangzhou Medical University (Guangzhou, China).

### Cell culture

All the cell lines used in the study were primarily obtained from American Type Culture Collection (Rockville, MD, USA). The cells were cultured at 37 °C with 5% CO_2_ according to the standard protocols, with DMEM-F12 containing 10% fetal bovine serum, penicillin (100 U/ml) and streptomycin sulfate (100 µg/ml).

### MiRNAs and transfection

MiR-622 mimics (miR-622), its negative control (miR-control), the inhibitor of miR-622 and the inhibitor controls were obtained from RiboBio (Guangzhou, China). Lipofectamine 2000 (Invitrogen) was used for miRNAs or siRNA transfection.

### Cell proliferation

Kidney cancer cells were seeded in 6-well plates and transfected with miR-622 or miR-622 inhibitors or CCL18 and cultured in the normal condition. Cell survival ability was tested by the method of MTT (Sigma) assay.

### Dual luciferase reporter assay

CCL18 promoter activity was examined using Dual-Luciferase Reporter Assay System (Promega) according to the manufacturer’s instructions. Cells were seeded in 24-well plates and transfected the CCL18 3′UTR luciferase reporter, wild type or mutant reporter constructs and Renilla plasmid by using lipofectamine 2000 (Invitrogen). Luciferase activity were performed 48 h post-transfection using the Dual Luciferase Assay System (Promega, WI).

### Migration and invasion assay

Cell migration was determined using wound healing. RCC cells (1.0 × 10^4^) were transfected with CCL18 siRNA or miR-622 inhibitors for 24 h, and then seeded in the 12-well plate and observed the wound width. RCC cells were transfected with CCL18 siRNA or miR-622 inhibitors for 24 h, and then seeded in the up-chamber of the transwell system, the invaded cells underside of the membrane were counted.

### RNA extraction and real-time PCR analysis

Kidney cancer cells were transfected with miR-622 inhibitors or CCL18 siRNA or the controls for 48 h and then total RNA was isolated for RT-PCR analysis. The expression level of miRNAs was defined based on the threshold cycle (Ct), and relative expression levels were calculated using the 2^−ΔΔCt^ method, using the expression level of the U6 snRNA as a reference gene.

### Western blotting

Cultured cells were harvested and lysed with RIPA buffer containing the protease inhibitors on ice for 30 min. Protein were separated by SDS-PAGE. The protein was transferred onto nitrocellulose membrane using and probed with primary antibodies including phos-Erk, Erk, phos-p38, p38, phos-JUK, JUK, cdc25, CREB, Mad1, c-Fos and β-actin and then horseradish peroxidase-labeled secondary antibodies. All the antibodies were purchased from cell signaling technology. The protein band signals were visualized using an ECL.

### Statistical analysis

All analysis were performed using the SPSS 18.0 (SPSS, Chicago, IL, USA) or Excel. Every experiment was completed independently at least three times. A P < 0.05 was considered significant.

## Results

### Down-regulation of miR-622 in RCC tissues is correlated with clinicopathological characteristics

The expression of miR-622 was examined in RCC cells lines (769-P, A498, 786-O, GRC-1, OS-RC-2, ACHN) and normal kidney cells (HK-2) and miR-622 expression in the RCC cell lines was lower than its expression in HK-2 cells (Fig. 1a). The cell invasion was assayed by transwell system, and the data indicated that miR-622 could inhibited RCC cell invasion, but not in HK-2 cells (Fig. 1b). Furthermore, miR-622 expression was verified in the RCC tissues and exhibited extraordinarily low expression of miR-622 compared to the adjacent tissues (Fig. 1c). We divided the 112 patients with RCC into two groups: high metastasis (n = 78) and low metastasis including no metastasis (n = 34). We found that miR-622 expression in the RCC with high metastasis was lower than it in the RCC with low metastasis or without metastasis (Fig. 1d).

**Fig. 1:** Down-regulation of miR-622 in RCC tissues is correlated with clinicopathological characteristics. **a** miR-622 expression was measured in kidney cancer cells by RT-PCR. **b** The RCC cells and HK-2 cell invasion was assayed by transwell system. All the cells were transfected with miR-622 mimics and its control for 24 h and then seeded in the up-chamber with matrigel treatment. The cell invaded cells were counted under the microscope. **c** miR-622 expression was measured in RCC tissues by RT-PCR. **d** miR-622 expression in high metastasis (n = 78) and low metastasis (n = 34) of RCC. **P < 0.01; *P < 0.05

### MiR-622 is methylated in RCC cells

Some tumor suppressor miRNAs have been reported to be silenced by aberrant DNA hypermethylation. We therefore investigated the mechanisms whereby miR-622 functions in RCC cells, with an emphasis on epigenetics. We determined if miR-622 expression was silenced by DNA methylation by examining the reactivation of miR-622 expression in GRC-1, OS-RC-2, ACHN and HK-2 cells following treatment with the demethylating agent 5-aza. MiR-622 expression levels recovered by 3–5-folds after 5-aza treatment in GRC-1, OS-RC-2 and ACHN cells, but not HK-2 cells (Fig. 2a). Furthermore, we detected CpG island methylation of miR-622 in RCC cell lines (including 769-P, A498, 786-O, GRC-1, OS-RC-2 and ACHN) by BSP analysis of multiple clones in the cell lines. Bisulfite sequencing in all the above RCC cell lines confirmed marked methylation of the promoter region of miR-622, however, there was no methylation in normal cells (HK-2) (Fig. 2b).

**Fig. 2:** MiR-622 is methylated in RCC cells. **a** miR-622 expression in RCC and HK-2 cells following treatment with the demethylating agent 5-aza. **b** CpG island methylation of miR-622 in RCC cell lines and normal kidney epithelial cells (HK-2) by BSP analysis of multiple clones in the cell lines. **P < 0.01

### CCL18 is a the potential target gene of miR-622

It was predicted that CCL18 is the target gene of miR-622 by TargetScan 7.0 (Fig. 3a). We want to know whether miR-622 regulates CCL18 expression in OS-RC-2 and ACHN cells. MiR-622 were effectively down-regulated in OS-RC-2 and ACHN cells with miR-622 mimics or inhibitors transfection. We used RT-PCR to verify the most potential target genes and found that CCL18 mRNA was significantly down-regulated in OS-RC-2 and ACHN cells (Fig. 3b). CCL18 mRNA was significantly up-regulated in OS-RC-2 and ACHN cells with miR-622 inhibitors (Fig. 3c). The result was confirmed by ELISA (Fig. 3d, e). The luciferase assay was used to test whether CCL18 is the target gene of miR-622, and the results showed that luciferase activity in OS-RC-2 and ACHN cells was down-regulated significantly when the cells were co-transfected with miR-622 mimics and wide type of CCL18 3′UTR (Fig. 3f). It was also verified that the luciferase activity in OS-RC-2 and ACHN cells increased significantly when the cells were co-transfected with miR-622 inhibitors and wide type of CCL18 3′UTR (Fig. 3g).

**Fig. 3:** CCL18 is a potential target gene of miR-622. **a** The predicted result from targetscan. **b** MiR-622 mRNA levels in OS-RC-2 and ACHN cells. OS-RC-2 and ACHN cells were transfected with miR-622 mimics for 48 h and RNA was extracted for RT-PCR. **c** MiR-622 mRNA levels OS-RC-2 and ACHN cells. OS-RC-2 and ACHN cells were transfected with miR-622 inhibitors for 48 h and RNA was extracted for RT-PCR. **d** CCL18 protein levels in OS-RC-2 and ACHN cells with miR-622 mimics transfection were texted by ELISA. **e** CCL18 protein levels in OS-RC-2 and ACHN cells with miR-622 inhibitors transfection were texted by ELISA. **f** Luciferase activity in 293T cells was down-regulated significantly when the cells were co-transfected with miR-622 mimics and wide type of CCL18 3′UTR. **g** Luciferase activity in 293T cells was down-regulated significantly when the cells were co-transfected with miR-622 inhibitors and wide type of CCL18 3′UTR. **P < 0.01

### MiR-622 suppresses kidney cancer cell survival and metastasis by targeting CCL18

To investigate the effect of miR-622 on RCC cell survival and metastasis ability, OS-RC-2 and ACHN cells were transfected with the mimics of miR-622 and treated with CCL18 (50 ng/ml) and cell proliferation was measured using MTT method. We found that OS-RC-2 cell growth was enhanced in cells with miR-622 overexpression and in CCL18 treated cells (Fig. 4a). There were similar results in ACHN cells (Fig. 4b). The result from the wound healing assay showed that miR-622 suppressed OS-RC-2 and ACHN cell migration stimulated with CCL18 (Fig. 4c–e) Transwell system was used to observe the cell invasion ability and the result showed that the invaded cells became less in the group of cells with miR-622 than the controls and miR-622 also decrease cell invasion of CCL18-overexpressed cancer cells (Fig. 4f–h).

**Fig. 4:** MiR-622 suppresses kidney cancer cell survival and metastasis by targeting CCL18. **a**, **b** OS-RC-2 and ACHN cells were transfected with the mimics of miR-622 and treated with CCL18 (50 ng/ml) and cell proliferation was measured using MTT method. **c** OS-RC-2 and ACHN cells were transfected with the mimics of miR-622 and treated with CCL18 (50 ng/ml) and cell invasion was measured using wound healing method. **d**, **e** Data from C were quantified. **f** OS-RC-2 and ACHN cells were transfected with the mimics of miR-622 and treated with CCL18 (50 ng/ml) and cell invasion was measured using transwell chamber. **g**, **h** Data from F were quantified. *P < 0.05; **P < 0.01

### MiR-622 has negative relationship with CCL18 in RCC tissues

To investigate the relationship between miR-622 expression and CCL18 levels in RCC tissues and cell lines, CCL18 expression in tissues of RCC patients were assayed by RT-PCR. The data showed that CCL18 mRNA levels were enhanced in 112 RCC samples than the controls (Fig. 5a). MiR-622 expression in the tissues of 112 RCC patients were assayed by RT-PCR. The data showed that miR-622 expression was decreased in RCC samples than the controls (Fig. 5b). The analysis of relationship between miR-622 and CCL18 levels in the samples showed that both of them had negative association (Fig. 5c).

**Fig. 5:** MiR-622 has negative relationship with CCL18 in RCC tissues. **a** CCL18 mRNA expression in the tissues of RCC patients were assayed by RT-PCR. **b** MiR-622 expression in the tissues of RCC patients were assayed by RT-PCR. **c** The analysis of relationship between miR-622 and CCL18 mRNA levels in the samples. *P < 0.05; **P < 0.01

### MiR-622 inhibits CCL18 activated MAPK signal pathway in RCC cells

CCL18 could activate MAPK signal pathway. Whether miR-622 inhibits CCL18 mediated activated MAPK in RCC cells, OS-RC-2 and ACHN cells were transfected with miR-622 mimics or treated with CCL18 and then the molecules associated with MAPK signal pathway were detected. When the cells were treated with CCL18, Erk and JUK was phosphorylated, p38 was not influenced and miR-622 inhibited the activated Erk, however, p38 and JUK was not affected; miR-622 could suppress the protein levels of cdc25, CREB, c-Fos, Mad1 induced by CCL18 in OS-RC-2 and ACHN cells (Fig. 6a). The mRNA levels of MAPK associated proteins were measured and the data indicated that the mRNA of the genes involved in cell proliferation, metastasis associated MAPK signal pathway was enhanced in the OS-RC-2 and ACHN cells with CCL18 treatment, and miR-622 suppressed them (Fig. 6b, c).

**Fig. 6:** MiR-622 inhibits CCL18 activated MAPK signal pathway in OS-RC-2 and ACHN cells. **a** OS-RC-2 and ACHN cells were transfected with miR-622 mimics or treated with CCL18 and then the molecules associated with MAPK signal pathway were detected by western blotting. **b**, **c** OS-RC-2 and ACHN cells were transfected with miR-622 mimics or treated with CCL18 and the mRNA levels of cdc25, CREB, c-Fos, Mad1 were measured by RT-PCR. *P < 0.05; **P < 0.01

## Discussion

It is very common for the dysregulation of miRNA expression in RCC. In cancer development and progression, miR-622 plays as a tumor inhibitor or an oncogene. MiR-622 plays an inhibiting role in glioma cell proliferation, invasion and migration by down-regulating transcription factor 2 [7]. MiR-622 suppresses migration and invasion by targeting DYRK2 in colorectal cancer cells [9]. MiR-622 acts as a tumor suppressor in colorectal cancer occurrence and metastasis by suppressing K-Ras [10], in hepatocellular carcinoma [12], in lung cancer by repressing hypoxia-inducible factor-1α in ERK-responsive [13], in human esophageal squamous cell carcinoma by directly targeting E2F1 [14], in gastric cancer by targeting LAMC2 and CD82 [15]. However, in some conditions, miR-622 plays an oncogene, for example, radiation could increase miR-622 expression and then promotes radioresistance of colorectal cancer cells by targeting Rb expression [8]. In RCC, the functional roles of miR-622 were not known. In this study, we found that low levels of miR-622 in RCC tissues and cells, which suppressed cell proliferation and metastasis by targeting CCL18 expression.

Some of the aberrant miRNAs were methylated. Hypermethylation of CpG islands is known to be an epigenetic modification. Dysregulation of miRNAs can be caused by epigenetic modifications, including DNA methylation and the covalent modification of histone protein, which do not directly change the DNA sequence. Methylation of CpG islands in the gene promoter has been strongly linked to the silence of tumor-suppressor gene expression in cancer. Several tumor-associated miRNAs have been reported to be silenced by aberrant hypermethylation of their promoter regions in various cancers, including miR-9, miR-137, miR-127, miR-34b/c, miR-148, miR-342, and miR-127 [16–19]. Our study showed that the expression of miR-622 in RCC tissues samples of patients with RCC was lower than the normal controls. Its expression is restored by 5-aza-dC treatment, suggesting that abnormal expression of miR-622 is epigenetically regulated due to DNA hypermethylation RCC cells. Based on expression analysis of miR-622 in RCC cell lines treated with 5-aza, we strongly suspected that DNA methylation was one of the regulatory mechanisms of miR-622 expression. In order to confirm the DNA methylation associated with abnormal expression of miR-622, bisulfite sequencing analysis was performed to assess the methylation status of CpG islands of miR-622, and we observed that miR-622 was hypermethylated in RCC cell lines.

CCL18 plays important roles in cancer progression and its expression was regulated by miRNAs. It is reported that miR-181b inhibits CCL18-induced breast cancer cell metastasis and invasion via the NF-κB signaling pathway [20]. Let-7a mimic attenuates CCL18 induced breast cancer cell metastasis through Lin 28 pathway [21]. CCL18-mediated down-regulation of miR98 and miR27b promotes breast cancer metastasis [21]. Our functional analyses described that miR-622 suppressed cell growth, migration, and invasion, demonstrating that miR-622 acted as a tumor suppressor. In our study, we showed that miR-622 reduced the expression level of CCL18 at both mRNA and protein levels in RCC cells. The luciferase activity assay with a reporter containing the miR-622 binding sequence at the 3′ UTR of mRNA suggested that miR-622 directly targets the 3′ UTR of CCL18 mRNA.

In summary, our results indicated that aberrant expression of miR-622 was regulated by DNA hypermethylation in RCC. Functional analysis suggested that miR-622 suppresses RCC cell growth and metastasis by targeting CCL18. Overall, all of these data suggest that miR-622 might play a role as tumor suppressor in RCC.

## Conclusions

The study demonstrated that CCL18 was a target gene of miR-622 in kidney cancer cells, which was from the prediction result. The clinical results demonstrated that miR-622 was negatively associated with CCL18 in the samples of RCC patients. The further investigation indicated that miR-622 suppressed CCL18 activated MAPK signal pathway in RCC cells.
